The article "The Influence of Network Location on Knowledge Hiding from the Perspective of Lifelong Education" was retracted in 2023. Reasons: unreliable results or conclusions; concerns about the data; concerns about the results or conclusions; concerns about the peer review.

# The Influence of Network Location on Knowledge Hiding from the Perspective of Lifelong Education

**DOI:** 10.1155/2022/4881775

**Published:** 2022-08-30

**Authors:** Huan Liu, Mingfang Dong

**Affiliations:** ^1^School of Economics and Management, Northwest University, Xi'an 710127, China; ^2^School of Management, Xi'an University of Architecture & Technology, Xi'an 710055, China

## Abstract

Inhibiting negative knowledge behavior is one of the ways to improve the effective circulation of knowledge within the organization. This study puts employees' knowledge hiding behavior in the organizational relationship network situation and discusses the influence of network location on knowledge hiding, exploring the moderating role of knowledge acquisition in the relationship between network location and knowledge hiding. From the perspective of social network, 232 knowledge-based employees were used to obtain the data, and we used literature analysis, social network analysis, multiple regression analysis, UCINET, SPSS, and other software packages. Research shows that employees in the central network are less willing to do knowledge hiding behavior, and those in the structural hole network tend to do knowledge hiding behavior. Knowledge acquisition as the supply way of knowledge resources plays a positive role on the negative relationship between centrality and knowledge hiding and on the positive relationship between structure hole and knowledge hiding. The research results have positive significance for understanding and mastering the hiding behavior law of individual knowledge in the organizational relationship network and also provide certain theoretical basis and data support for organizational knowledge governance.

## 1. Introduction

The World Organization for Economic Cooperation and Development recognized as early as 1996 that knowledge and technology have become the driving force of productivity and economic growth in the modern economy. The new focus of economic performance is on knowledge, technology, and learning. Unlike the use of rare resources in the early economy, knowledge is not only a resource that will not dry up after use but also the value of knowledge increases in the transmission and transfer. Knowledge sharing is an effective way to promote knowledge transmission and transfer. Although organizational managers have made great efforts to promote employee knowledge sharing behavior, it is difficult to achieve effective knowledge sharing among employees within the organization. This is because the organization is not the owner of the individual knowledge assets of the employees and cannot force or forcibly implement knowledge sharing and can only take certain incentive measures and reasonable rules or regulations to promote knowledge sharing. In recent years, many scholars advocate that corresponding management measures can be taken to restrain a series of negative knowledge behaviors that hinder employees from the perspective of reverse, which may have an unexpected effect on promoting knowledge sharing within the organization.

Knowledge hiding is a negative knowledge behavior that has been confirmed [1]. It negatively affects the sharing, dissemination, and innovation of knowledge within the organization through organizations, interpersonal relationships, and individual employees, such as Cerne et al. suggested that knowledge hiding reduces individual creativity levels [2] and employee innovative behaviors [3], and it can also affect individual performance. There is also evidence that knowledge hiding can be disseminated from managers to followers [4]; knowledge hiding increases the high levels of distrust and competitiveness [5]. In 2012, Connelly and other scholars clearly defined the concept of knowledge hiding [6], and then, scholars carried out a series of studies on the occurrence mechanism and consequences of knowledge hiding behavior, which further expanded our understanding of knowledge transmission mechanism in organizations, and had an important impact on the successful implementation of knowledge management in enterprises [7]. Based on the existing research results, the occurrence mechanism of this behavior is still in the early stage of exploration, and the pre-dependent variables affecting employee knowledge hiding behaviors need to be studied in depth. Compared with the complicated organizational situation, the relevant research still needs to be improved and excavated. Especially for knowledge employees as knowledge carriers, they are embedded in complex social relations and connection networks, and the flow of knowledge between organizations will inevitably be affected by the structure of the relationship network. However, so far, few scholars have discussed the causes of network location on individual knowledge hiding behavior from the perspective of social network. Due to the complexity of social networks and the sociability of knowledge hiding behaviors, the influence of network structure on knowledge hiding behaviors cannot be ignored, and different employees in different network positions can acquire knowledge and have different knowledge values. Some positions play a key role in knowledge transmission, and some positions become the center of knowledge circulation. Based on the above analysis, this study mainly focuses on the following two issues:

  Will employees influence their knowledge hiding behavior due to their different network locations in the network within the organization?
  If in the same network position, will employees affect the degree of hidden knowledge by how they acquire knowledge?

In conclusion, this study starts from the perspective of social network, takes knowledge-based employees as the research object, and verifies the hypothesis model through empirical analysis, to explore the influence mechanism of network location on employee knowledge hiding behaviors. The research results not only enrich the discussion of the dependent variables before employee knowledge hiding behaviors but also improve the research on the occurrence mechanism of employee knowledge hiding behaviors and further expand the understanding and understanding of the knowledge transmission mechanism in the organization [8]. It provides certain theoretical basis and data support for the management activities and staff knowledge management in the organization, formulates a more perfect management system to better release the knowledge resources in the organization, and promotes the effective flow and innovation of knowledge resources.

## 2. Concept Definition and Literature Review

As a key variable in social network analysis, network location is the result of the complex relationships of social networks among actors [8]. Nodes in different positions have different location advantages. Burt believes that the diversity of backgrounds and experiences of network members provides multiple knowledge for businesses [9]. Casper believes that if enterprises occupy a good network position, they will have a high reputation, which will attract more network members to establish relationships with them, and will continue to have the advantages of information source and processing [8]. There are many variables to measure the network location, but the main variables widely studied and best reflect the network location are the centrality [10] and structural hole [11]. Qian Xihong et al. study the impact of network location on innovation activity by dividing it into two dimensions: centrality and structural holes [12]. In the research of technological innovation network, Yang Yi et al. also measured the network structure through the two dimensions of centrality and structural hole [13]. In collaborative innovation networks, different network locations represent different opportunities to acquire new knowledge [14]. Accordingly, the network location plays a vital role in the acquisition and flow of internal and external knowledge in the organization.

Burt believes that the core degree of information exchange in the network structure is measured by centrality, including the strength of individual contact with others and the frequency of information communication. The centrality emphasizes the characteristics of a direct connection to the self [15]. Wasserman and Galaskiewicz (1984) proposed that centrality considers the degree of individual access and control of resources [16]. The high degree of centrality indicates that the individual is at the core of the organizational network, has greater influence and visibility [17], and also has wider connections, and other members of the organization network achieve greater willingness and more opportunities for knowledge sharing. The low centrality indicates that the individual is on the edge of the organizational network and has a low intensity of contact with others and resource control. Structural holes differ from centrality concerns, and structural holes emphasize the properties of heterogeneous connections. Burt (1992) uses structural holes to represent nonredundant connections, arguing that “nonredundant contacts are connected by structural holes” [18], measuring individual control over these nonredundant resources and information. The structural hole builds a “bridge” for many other individuals or organizations that have no connection, then opens up the channels of various heterogeneous information and resources, and promotes the flow and innovation of information and knowledge. By controlling the flow of information and resources between other nodes, actors who occupy structural holes on the one hand enrich their own information resources and on the other hand have more information sources and processing advantages because of controlling the lifeblood of resources. Burt believes that the structure of structural hole can provide nonredundant knowledge and information for individuals in this position, improve their competitiveness, and thus bring themselves advantages such as fame, promotion, and salary increase [19]. Studies have confirmed that network location (centrality, structure hole) has an important impact on the acquisition, sharing, and flow of knowledge resources within the organization, but it has not demonstrated the impact of network location on the negative knowledge behavior of employees' knowledge hiding. Although scholars Hongdan Zhao and Jiarui Jiang based on the social network perspective in the study of knowledge hiding behaviors introduced the structure hole and center of these two variables, but only discussed the center and structure hole that jointly regulate the role of stress on emotional exhaustion and the indirect effect of hidden knowledge [20], it did not directly explore the influence of center and structure hole for knowledge hiding behaviors. This study considers the influence of network location through the variables of center degree and structure hole.

In the era of knowledge economy, the depreciation of human capital caused by employees' failure to timely acquire and update their knowledge and skills has become a key factor affecting the development of individual employees and organizations. Continuous knowledge acquisition ability has become the power source of lifelong learning of knowledge-based employees and also the necessary lifelong learning ability of knowledge-based employees. Therefore, as an important basis for knowledge management in the lifelong learning situation of a knowledge-based organization, knowledge acquisition is increasingly receiving widespread attention. Huber knowledge acquisition is considered as the “process of knowledge acquisition,” which refers to the behavior of individual employees to acquire organizational knowledge and other knowledge [21]. Harem et al. (1996) believe that knowledge acquisition refers to the process of cognition and knowledge transfer of the same knowledge receiver [22]. Management master Peter Drucker believed that the distinction between manual workers and knowledge workers grew as the workplace changed. Handworkers use their hands to create products and services, while knowledge workers use their minds to create ideas, information, and knowledge that can add value to the company. Therefore, for knowledge-based employees, only by continuously acquiring external knowledge they can make up for their own knowledge stock and their quality shortage [23] and obtain personal competitive advantage [24]. As the carrier of knowledge, only by constantly acquiring themselves and external knowledge they can realize the supplement and reserve of knowledge resources, thus producing different learning and behavioral consequences and realizing value-added goals. Knowledge acquisition means the sharing and integration of more cutting-edge theories and different perspectives. It helps employees to get more innovative inspiration and accelerate the generation of innovative behavior [25]; Drees and Heugens believe that knowledge acquisition can continuously meet the needs of innovation [26]; Svec Vlastimil et al. discuss the the implicit knowledge acquisition of managers [27]; although previous studies have affirmed the positive impact of knowledge acquisition on organizational and individual knowledge innovation and competitive advantage, it also makes it clear that the different knowledge acquisition behaviors of employees directly affect the acquisition efficiency and quality of the diffusion from the knowledge source to the knowledge recipient, but very few studies have explored the relationship between knowledge acquisition and negative knowledge behavior. There are also few studies that employees employee knowledge acquisition behavior in a complex network context. Therefore, based on the perspective of social network relations, this study will explore whether individual employees' attitudes towards knowledge hidden behaviors are affected by knowledge acquisition when they encounter knowledge requesters seeking some knowledge from themselves.

In 2012, Connelly and other scholars called knowledge hiding of individuals in organizations to face knowledge requests from colleagues [6]. The knowledge hiding is further divided into three dimensions: evasive hiding, playing dumb, and reasonable hiding. Knowledge hiding is proven to be a negative behavior in the workplace [28], and knowledge hiding is just beginning compared with the emphasis on knowledge sharing in human resource management research. Existing research evidence suggests that knowledge hiding reduces individual and team creativity, reduces individuals' innovative work behavior, and increases voluntary turnover. Although organizations implement various incentives to promote knowledge sharing, knowledge-sharing initiatives do not necessarily eliminate knowledge hiding because there are different drivers of knowledge hiding; e.g., from a leadership perspective, Donate Mario J and other scholars found that knowledge-oriented leadership has a positive and strong direct impact on knowledge hiding [29]; Agarwal Upasna et al confirmed that ethical leadership can reduce the occurrence of knowledge hiding behaviors [30]; Changyu Wang and other scholars confirmed that the abusive management implemented by leaders has a positive impact on subordinates' knowledge hiding behaviors [31]; Yuan Ling et al. verified that the U-type curve relationship between humble leadership and employee knowledge hiding was significant [32]; from the perspective of knowledge attributes, scholars such as Sulistiawan Jovi have confirmed that knowledge complexity is also an important factor affecting employees' knowledge hiding; from the perspective of individual characteristics, Soral Prakriti and others believe that the dark personality traits of superiors will enhance the knowledge hiding behaviors of subordinates [33]; Zoe Geofroy and Max Evans believe that employees with high emotional intelligence are less likely to hide their knowledge [34]; from the perspective of the organizational atmosphere, Oubrich Mourad et al.'s studies have confirmed that organizational equity reduces the occurrence of knowledge hiding behavior within organizations [35]; Li Hao et al. have verified that defense orientation has a promoting effect on knowledge hiding in enterprises, performance atmosphere can enhance the impact of defense orientation on knowledge hiding, and the adjustment effect of weak performance atmosphere and strong performance atmosphere changes with the change in defense orientation [36]; from the perspective of interpersonal relationships, scholars such as Sulistiawan Jovi have confirmed that interpersonal distrust is a key factor in predicting employee knowledge hiding [37]; Cheng and Bao explored the promotion of negative rumors among employees in knowledge hiding [38]; Cegarra-Navarro Juan-Gabriel and other scholars found that defensive practices produced by interpersonal relationship were positively correlated with knowledge hiding [39]; Alam Tahira and other scholars found that relationship conflict positively affects knowledge hiding [40]; Sidra Riaz et al. studies have confirmed that workplace exclusion positively influences knowledge hiding behavior [41]; Connelly and Zweig will be the interpersonal deterioration [42]. The organization network of the individual cannot be ignored. It is worth exploring whether the unique network location of the organization network relationship affects the knowledge hiding behavior of the employees.

## 3. Study Assumptions

### 3.1. Centrality and Knowledge Hiding

Social network theory holds that social networks are a collection of social actors acting as nodes and the relationships between them [43]. Actors are interdependent rather than independent individuals. Their association is the channel of resource transfer or “flow.” Each individual in the network structure has its own field and location according to its own resources. It is located in nodes at different locations and has different location advantages. Individuals with advantageous positions are more likely to access new information and knowledge from different locations. The central location is a special position with greater attraction and visibility; because of its central position, it can share more common information and knowledge with other members. Bavelas' groundbreaking hypothesis in 1950 was that the closer an individual gets to the center of the network structure, the more impact it has [44]. Sparrowe (2001) believes that the higher the center of the individual in the network structure, the more comprehensive the information they have, and the higher their ability to deal with problems [45]. In addition, Chang Hongjin et al. believe that enterprises in central positions are more likely to form stable relationships with enterprises in other positions, be perceived with higher credibility, and reject other possible options [46]; based on the principle of indirect reciprocity, employees will show more altruistic and helpful prosocial interests to better establish relationships and maintain and consolidate interpersonal connections, thus promoting the occurrence of employee cooperative behaviors. Therefore, we believe that the members of the organization located in the structural center of the organization network are more willing to share their knowledge and expand and consolidate their influence, rather than hiding their knowledge. Therefore, the hypothesis is that there is a negative correlation between centrality and knowledge hiding.

  H1: there is a negative correlation between centrality and knowledge hiding; according to the theory of social capital, in an organizational structure, the higher the individual uses his special position, the higher his social capital. The higher the social capital will consolidate his central position, become the trusted object of other members of the organization, and continue to be attractive. Therefore, constantly acquiring new knowledge can more reflect the value of the central position members and therefore does not retain the knowledge requests of other members. We conclude that we hypothesize that knowledge acquisition has a reinforcing role in the negative correlation between centrality and knowledge hiding as follows.
  H2: knowledge acquisition has a positive regulatory effect on the relationship between centrality and knowledge hiding.

### 3.2. Structural Hole and Knowledge Hiding

Employees who occupy the structural hole can approach much different information flow and knowledge flow, obtain many nonredundant knowledge resources, and form information advantage; the structural hole can obtain “information benefit” and “control benefit” opportunities [47], thus bringing competitive advantages such as job promotion, salary increase, or reputation, and the more obvious the individual advantage with more structural holes. The theory of territorial behavior believed that the territorial behavior exists widely in the organization, which is the behavioral expression of the psychological ownership perception of a certain target territory in the organization. When the territory is lost, the individual will experience a very strong psychological pressure and unpleasant feeling. To maintain the competitive advantage brought by the structural hole, individual employees consolidate their knowledge resources and reduce the possibility of losing knowledge territory. When others request knowledge from the knowledge owner in the position of the structural hole, the knowledge owner has a stronger motivation to hide knowledge. Thus, we introduce the hypothesis:

  H3: there is a positive correlation between the structural hole and the knowledge hiding; resource preservation theory holds that individuals have the basic motivation to acquire, maintain, and protect resources. Individual employees maintain and protect their knowledge and information and constantly consolidate and control their knowledge resources through knowledge acquisition to avoid the pressure arising from the loss of knowledge resources. For them, the potential or actual loss of knowledge resources is a threat. These knowledge resources can not only meet individual needs but also help employees to conduct accurate self-identification and social positioning [48]. The more precious resources are the more difficult to obtain, the more sensitive the individual is to their loss. Employees in the structural hole position have more access to nonredundant knowledge resources that are difficult to obtain by other members. With the continuous acquisition of knowledge resources, the employees in the structural hole position have the stronger motivation to prevent the loss of knowledge resources. To sum up, individuals will constantly enrich knowledge resources due to knowledge acquisition and then strengthen the positive relationship between structural holes and knowledge hiding. This introduces the hypothesis as follows.
  H4: knowledge acquisition has a positive regulatory effect on the relationship between structural hole and knowledge hiding; in conclusion, the theoretical model proposed in this study is shown in Figure 1.

## 4. Research Method

### 4.1. Study Design and Sample Collection

The respondents are mainly knowledge employees in knowledge-intensive positions. Since the measurement variables include social network structure variables, the questionnaire is divided into three parts: the second part is the traditional questionnaire mode, which makes the Likert 7-point scale measurement of knowledge hiding and knowledge acquisition variables, and the third part uses the nomination generation method to obtain the data of calculating centrality and structure hole. This method has high reliability and validity. At present, the proposed method has formed a set of mature processes and processing methods, which are quite widely used. We used a semi-open questionnaire to obtain employee contact. First, the list of knowledge team members is determined. To minimize the concerns of the subject, we code the member list; then, we ask the subject to select the team member code according to whether it is related at work; finally, the collected questionnaire is 0–1 for team members with 1 and 0. The combed questionnaire data form a standard 0–1 matrix; by importing the data in the matrix into the UCINET software, you can get the specific indicators of each team member about the centrality and the structure of the hole. The index data of centrality and structural holes were collated to provide data support for the later multiple regression analysis.

Due to the particularity of the third part, we mainly distributed the questionnaire by the internal knowledge team of the enterprise, which was filled in by the team members independently. In view of the difficulty of data collection, we mainly adopted the introduction of acquaintances and field visits and distributed and collected questionnaires through electronic media and on-site distribution. Either way, the respondent was explained in detail before the delivery, to ensure that each respondent understood the filling rules of the questionnaire and to minimize the concerns of the real-name questionnaire, so as to improve the quality and efficiency of the questionnaire distribution. Finally, 286 questionnaires were issued to 32 teams. After excluding invalid questionnaires, 232 valid questionnaires from 25 teams were finally obtained, and the effective recovery rate was 81.2%. Descriptive statistics of the sample are shown in Table 1.

### 4.2. Variable Measurement

The measurement variables of knowledge hiding and knowledge acquisition are both from the existing mature scale. In the Chinese context, the English scale was translated into the Chinese scale by combining Chinese and English translation and corrected according to the specific research objects and situations to ensure the reliability and validity of the study. Except for control variables, Likert 7-point scale ranged from “1” to “7” to represent “complete consent” to “complete consent.” The measurement of knowledge hidden variables uses a measurement scale developed by Connelly, including a total of “Suppose a colleague asks you for some important knowledge, you refuse his/her request, you may…,” “verbally promised to help him/her, but in fact I will not put into action,” and other 12 items. The knowledge acquisition variables draw on the mature scale developed by Wu Yong and others, including nine measurements such as “I often attend training sessions and seminars organized by the company” and “I often talk and listen honestly with colleagues.”

The network position is measured by centrality and structure hole, and the data are obtained by UCINET software. Where centrality is measured by degree centrality, the number of individuals is directly linked to the study individual. The greater the degree of an individual, the more the individual tends to be in a central position, and the more relationships with it. Structural holes are measured using the structural hole index given by Burt (1992) himself. Effective scale, efficiency, limit system, and hierarchy are the four indicators considered by structural holes, among which the third index is the most important; in this study, we measure the number of structural holes through the limit system. The high restriction index indicates that the number of individual structural holes is small. Sex, age, education, length of service, and corporate nature were identified as control variables.

### 4.3. Data Quality Inspection

#### 4.3.1. Homology Deviation

In this study, Harman's single factor detection method was used to test the uncontrollable homology error in knowledge hiding and knowledge acquisition. After exploratory factor analysis of all variables, a total of seven common factors have characteristic values greater than 1, which jointly explained 62.237% of the variance variation, with the maximum explanatory force being 13.123%, without the 40% limit. This result indicates that the homology bias is not obvious; that is, each factor is independent.

#### 4.3.2. Confidence Analysis

The reliability of knowledge hiding and knowledge acquisition indicators was analyzed by SPSS 22.0, using Cronbach's *α* and composite reliability coefficients to test whether the structure measured by the questionnaire data is true. Hair et al. have suggested that the series value should be above 0.7. After removing the measurement variables with lower factor load, the reliability coefficient of the remaining 10 measures in the questionnaire is 0.841, and the reliability coefficient of 9 measures was 0.872, and Cronbach's *α* of all factors is higher than 0.7. Given that the measurement index of each construct is greater than 1, the credibility of the questionnaire was further confirmed by the index value CR representing the internal consistency reliability quality, i.e., the combined reliability. When the combined reliability CR is above 0.70, it means that the latent variable has a good combined reliability. Through calculation, the combined reliability of knowledge hidden variable is 0.9331, and the combined reliability of knowledge acquisition variable is 0.9131, which met the adaptation criteria (as shown in Table 2). Therefore, the data collected by the questionnaire in this study are stable and credible.

#### 4.3.3. Validity Analysis

The validity test is also a measure for knowledge hiding and knowledge acquisition. Validity measurement term represents the extent to which measurement results correctly reflect the connotation of the variable. The measurement scales of this study are from mature scales in domestic and foreign literature, and we consult the opinions of practical and theoretical experts in the field of knowledge management and make appropriate modifications to ensure that the scale has high content validity. The validity of the questionnaire was further ensured by calculating the convergent validity AVE value. The larger the AVE value, the stronger the potential variable can explain the corresponding item at the same time, the stronger the ability to show the nature of the potential variable (convergence to a point), and the better the convergence validity. When the AVE value is greater than or equal to 0.50, the latent variable has good convergent validity. The results showed that the AVE value of knowledge hidden variable was 0.6423 and the AVE value of knowledge acquisition variable was 0.7013, both indicating that the measurement scale had good convergence validity (as shown in Table 2). The above calculation results show that the questionnaire has good reliability and validity and can be used for the structural equation model test.

In addition, the centrality and structural hole values were calculated using UCINET in strict accordance with the nomination generation procedure.

## 5. Empirical Analysis

### 5.1. Descriptive Statistics of the Variables

The mean values, standard deviation values, and correlation coefficients of each variable in this study are shown in Table 3. Therefore, employees have a significant negative correlation with knowledge hiding (*r* = −0.238, *p* < 0.05) and a significant positive correlation with knowledge hiding (*r* = 0.281, *p* < 0.05), which provide preliminary support for the hypothesis of this study and lay the foundation for further explaining the regression analysis of the degree of correlation and influence among the study variables.

Multiple regression analysis was used to test the study hypotheses and the theoretical model multicollinearity detection showed smaller VIF values for each model, indicating high reliability of model estimation results, namely, no significant collinearity problem between variables. The results of the multiple regression analysis are shown in Table 4. According to Table 4, the centrality has a significant negative influence on knowledge hiding, indicating that the more the employee is, the less the knowledge hiding behavior is. Hypothesis 1 holds; the structural hole has a significant positive effect on knowledge hiding, indicating that the more the employee is in the structural hole, the more they will avoid or retain the knowledge requests from other individuals, and hypothesis 3 holds.

### 5.2. Regulatory Effect Test of Knowledge Acquisition

Network structure (centrality and structure hole) as independent variables, knowledge hiding as dependent variable, and knowledge acquisition as regulatory variable are taken to do hierarchical regression analysis. The results of Table 5 show that knowledge acquisition mode plays a positive role in the influence of knowledge hiding and knowledge acquisition mode in the influence of structural holes on knowledge hiding, and hypothesis 4 is true. The regulatory maps are shown in Figures 2 and 3, respectively.

## 6. Conclusions and Enlightenment

### 6.1. Conclusion

Employees are the most important resource in the organization, and the behavior efficiency of employees directly affects the efficiency of organizational activities. Therefore, how to mobilize the enthusiasm of employees and play their creativity is of great significance in the organizational management practice. This study explores the impact of network location on employee knowledge concealment from the perspective of lifelong learning and introduces knowledge acquisition as a regulatory variable and introduces knowledge acquisition as a regulatory variable to further explore the influence mechanism of network location and knowledge hiding, in which the network location is reflected by two variables: centrality and structure hole. On the basis of theoretical modeling and empirical analysis, we should further understand and master the hidden behavior rules of individual knowledge in organizations, improve the ability to predict, control, and guide individual knowledge behavior of employees, and then provide basis for managers to know people and take good responsibilities and cultivate and use people scientifically.

First, the results confirm that knowledge employees will influence their knowledge hiding behavior due to their different network locations in the relationship network within the organization. Centrality has a significant negative effect on knowledge hiding, while structural holes have a significant positive effect on knowledge hiding. Different network locations characterize different opportunities individual employees face in accessing knowledge resources within the organization. Employees in the center of the network have a wider range of knowledge search and dissemination than other employees, thus making it easier to gain the trust of members in other network positions. When other members of the organization make knowledge requests, they prefer to share with other members rather than retain or refuse. Centrality degree has a significant negative influence on knowledge hiding. Employees located in the structural hole can capture a large amount of nonredundant knowledge and information due to their unique network location and also create more new opportunities and new knowledge to ensure their unique position advantages and power in the network. Employees located in the structural hole will not easily share their knowledge resources, especially in obtaining difficult or valuable ones. When other employees make knowledge requests to him, they will refuse or retain them, which is not conducive to the internal innovation and knowledge transfer of the organization.

Second, the results show that if they are in the same network position within the organization, employees will affect the degree of hidden knowledge due to different knowledge acquisition. Among them, knowledge acquisition plays a positive role in regulating the influence of centrality on knowledge hiding; knowledge acquisition plays a positive role in regulating the influence of structural hole on knowledge hiding. As a certain pre-dependent variable of knowledge hiding behavior, network structure affects the willingness and attitude of individual employees when making knowledge requests from other organization members due to their different positions. The strength of this willingness and attitude is affected by individual knowledge acquisition. With the strengthening of knowledge acquisition, central employees are more willing to share their knowledge, reduce knowledge hiding behavior, and gain the embodiment of their own value; the more knowledge resources, the less willing to share knowledge and adopt knowledge hiding behavior.

### 6.2. Research Enlightenment

This study explores the relationship between network location and knowledge hiding behavior based on a lifelong learning perspective. On the theoretical level, first is enriching with studies of knowledge-hidden prebehavioral dependent variables. To further understand and master the occurrence mechanism of employee knowledge hidden behavior, sharing is made; next is breaking through the binary relationship between the knowledge requester and the owner, placing subjects in a more complex and realistic interpersonal network, and expanding the study of the occurrence situation of knowledge hidden behavior. The results are more consistent with the characteristics of the individual complex behavior and organizational relationship network and promoted our cognition and understanding of the knowledge transmission mechanism in the organization; last, to explore the negative knowledge behavior of knowledge concealment from the perspective of lifelong learning, the research perspective of knowledge hidden theory is enriched more; at the practical level, first of all, through the discussion of the dependent variables before knowledge hiding behaviors, we improve the managers' grasp of the occurrence law of employee knowledge hiding behaviors, then formulate corresponding management strategies, effectively inhibit the occurrence of knowledge hiding behaviors, and promote the effective flow and sharing of knowledge resources within the organization.

The study found that different network locations where employees are in organizational relationships have an impact on knowledge hiding behavior. Employees in centrality positions are less prone to knowledge hiding behavior. Managers can use the central employees as a hub for the effective circulation of knowledge resources within the organization. The occurrence of employee knowledge sharing behavior is stimulated by setting up benchmarking, training, and other mechanism measures. The conclusion is that employees in structural holes are more likely to have knowledge hiding behavior. Organization managers can use electronic media and OA office system to break down the knowledge barriers of employee knowledge, promote the flow of knowledge among staff-employees and staff-organizations, and the occurrence of employee knowledge hiding behaviors; next, knowledge acquisition plays a certain role in regulating the relationship between network location and knowledge hiding. In the negative relationship between knowledge acquisition and knowledge hiding, managers can enhance knowledge access to central employees, for example, professional training, the improvement of learning ability, drainage of more abundant knowledge resources to the central location of the employees, promoting the effective circulation of organizational knowledge resources; in the positive relationship between structural hole and knowledge hiding, on the one hand, managers can weaken the knowledge input of employees in the structural hole through task design, job adjustment, and other measures. On the other hand, the input of knowledge resources for other employees can also be increased by increasing training and electronic media, weakening the network structure and position of employees, and suppressing the occurrence of employee knowledge hiding behaviors.

### 6.3. Research Limitations and Outlook

This study has made some theoretical progress through theoretical modeling, questionnaire survey, and data analysis, but there are still many limitations.

First, the measurement of the network structure has some limitations. Thus, it is possible to bias the study, further strengthen the training of research personnel in the future, and reduce this deviation as much as possible; second, this study as a whole measurement and analysis did not study the detailed dimensions, although the scale effectively measures the knowledge hiding behaviors, to develop more detailed and accurate management strategy, the future we can try to knowledge hidden into different dimensions and explore the causes and consequences of knowledge hiding behaviors; thirdly, it is about the definition of knowledge type; how to suppress knowledge concealment behavior and stimulate organizational knowledge sharing has always been an important proposition of organizational knowledge management. At present, the academic circle divides knowledge into explicit knowledge and implicit knowledge according to the degree of knowledge transferability. Compared with simple and easy-to-transfer explicit knowledge, individuals tend to hide complex and difficult knowledge to transfer explicit knowledge. This study does not distinguish between the types of organizational knowledge, and whether explicit knowledge and implicit knowledge are different in the hidden behavior occurrence mechanism of employee knowledge is a question of further attention. In addition, how to make explicit the tacit knowledge to reduce the difficulty of knowledge transfer, promote the effective flow of knowledge within the organization, and reduce the negative impact of knowledge hiding among employees is also the issue that we need to focus on.

Finally, the research object of this article is limited to the staff level, although the study in complex organization relationship network situation for knowledge hiding behaviors opens up a new vision, influence knowledge is hidden before many variables, worth our deeper step of exploration and perfect; later, we organize internal cross-level research, and this is also a research direction in the future.

## Figures and Tables

**Figure 1:** Theoretical model.

**Figure 2:** Schematic diagram of centrality.

**Figure 3:** Schematic diagram of structure hole.

**Table 1:** Samples describing the statistical distribution.

Project	Class	Proportion (%)	Project	Class	Proportion (%)
Sex	Man	42.7	Record of formal schooling	High school and below	4.3
	Woman	57 3		Junior college	12 9

Age	Under 25	53.4		Undergraduate course	75.9
	25–35 years old	26.7		Master's degree or above	6.9
	36–45 years old	5.2		State-owned enterprises	32.3
	Over 45 years old	14.7	Enterprise nature	Foreign-owned enterprise	5.6

Length of service	Under 3 years	27.6		Private enterprise	34.5
	3–5 years	30 6		Other	27 6
	6–10 years	22.4			
	More than 10 years	19 4			

**Table 2:** Results of the reliability and validity tests.

Variable	Number of terms	Factor loading	Cronbach's *α*	AVE	CR
Knowledge acquisition	9	0.870	0.872	0.7013	0.9131
		0.895			
		0.894			
		0.827			
		0.713			
		0.858			
		0.844			
		0.763			
		0.820			
		0.700			
		0.827			
		0.769			
		0.752			

Knowledge hiding	10	0.777	0.841	0.6423	0.9331
		0.765			
		0.712			
		0.842			
		0.767			
		0.712			

**Table 3:** Descriptive statistical analysis table of the variables.

Variable	1	2	3	4	5	6	7	8	9
Sex									
Age	−0.317^*∗∗*^								
Record of formal schooling	−0.052	−0.284^*∗∗*^							
Length of service	−0.264^*∗∗*^	0.715^*∗∗*^	−0.207^*∗∗*^						
Position	−0.154^*∗*^	−0.042	0.216^*∗∗*^	0.172^*∗∗*^					
Industry type	0.083	0.295^*∗∗*^	−0.070	0.088	−0.500^*∗∗*^				
Central	0.118	−0.086	−0.061	−0.072	0.046	−0.090			
Structure hole	0.131^*∗*^	0.082	−0.005	0.037	−0.028	−0.068	−0.017		
Knowledge hiding	−0.39	0.220^*∗∗*^	0.014	0.178^*∗∗*^	0.086	−0.033	−0.238^*∗∗*^	0.281^*∗∗*^	
Average value (M)	1.57	1.81	2.85	2.34	2.15	2.96	0.6625	0.3292	3.4103
Standard value (SD)	0.496	1.068	0.592	1.081	1.191	1.815	0.24100	0.29639	1.06119

**Table 4:** Results of the multiple regression analysis.

Model	Argument	Knowledge hidden	
		Model 1	Model 2
	Constant		
	Sex	0.075	0.049
	Age	0.30^*∗∗*^	0.230^*∗*^
	Record of formal schooling	0.091	0.05
	Length of service	0.005	0.004
	Industry type	−0.102	−0.068
1	Central		−0.226^*∗∗∗*^
2	Structure hole		0.250^*∗∗∗*^
	F	2.462^*∗*^	5.514^*∗∗∗*^
	R2	0.071	0.183
	ΔR2	0.042	0.150

Note: ^*∗*^means *p* < 0.05, ^*∗∗*^means *p* < 0.01, and ^*∗∗∗*^means *p* < 0.001.

**Table 5:** Results of the regulatory effect test.

	Model 3	Model 4	Model 5	Model 6	Model 7	Model 8
Constant						
Sex	0.08	0.11		0.08	0.03	0.01
Age	0.30^∗∗^	0.29^∗∗^		0.30^*∗∗∗*^	0.24^*∗*^	0.26^*∗*^
Record of formal schooling	0.09	0.06		0.09	0.07	0.09
Length of service	0.01	−0.01		0.01	0.01	−0.01
Industry type	−0.10	−0.12		−0.10	−0.05	−0.06
Centrality		−0.23^*∗∗∗*^	0.24^*∗∗∗*^			
Knowledge acquisition		−0.06	−0.08			
Interactive item 1			0.28^*∗∗∗*^			
Structure hole					0.25^*∗∗∗*^	−0.24^*∗∗∗*^
Knowledge acquisition					−0.04	−0.04
Interactive item 2						0.15^*∗*^
*F*	2.46^*∗*^	3.62^*∗∗∗*^	5.60^*∗∗∗*^	2.46^*∗*^	3.86^*∗∗∗*^	4.12^*∗∗∗*^
*R* ^2^	0.07	0.13	0.20	0.07	0.14	0.16
Δ*R*^2^	0.04	0.09	0.17	0.04	0.10	0.12

## Data Availability

The data used to support the findings of this study are available from the corresponding author upon request.
